The article "Expedite Quantification of Landslides Using Wireless Sensors and Artificial Intelligence for Data Controlling Practices" was published in 2022. Journal: Comput Intell Neurosci.

# Expedite Quantification of Landslides Using Wireless Sensors and Artificial Intelligence for Data Controlling Practices

**DOI:** 10.1155/2022/3211512

**Published:** 2022-05-23

**Authors:** Pravin R. Kshirsagar, Hariprasath Manoharan, Samir Kasim, Asif Irshad Khan, Md Mottahir Alam, Yoosef B. Abushark, Worku Abera

**Affiliations:** ^1^Department of Artificial Intelligence, G.H Raisoni College of Engineering, Nagpur, India; ^2^Department of Electronics and Communication Engineering, Panimalar Institute of Technology, Poonamallee, Chennai, India; ^3^Department of Electrical and Computer Engineering, Faculty of Engineering, King Abdulaziz University, Jeddah 21589, Saudi Arabia; ^4^Computer Science Department, Faculty of Computing and Information Technology, King Abdulaziz University, Jeddah 21589, Saudi Arabia; ^5^Department of Food Process Engineering, College of Engineering and Technology, Wolkite University, Wolkite, Ethiopia

## Abstract

The power of wireless network sensor technologies has enabled the development of large-scale in-house monitoring systems. The sensor may play a big part in landslide forecasting where the sensor linked to the WLAN protocol can usefully map, detect, analyze, and predict landslide distant areas, etc. A wireless sensor network comprises autonomous sensors geographically dispersed for monitoring physical or environmental variables, comprising temperature, sound, pressure, etc. This remote management service contains a monitoring system with more information and helps the user grasp the problem and work hard when WSN is a catastrophic event tracking prospect. This paper illustrates the effectiveness of Wireless Sensor Networks (WSN) and artificial intelligence (AI) algorithms (i.e., Logistic Regression) for landslide monitoring in real-time. The WSN system monitors landslide causative factors such as precipitation, Earth moisture, pore-water-pressure (PWP), and motion in real-time. The problems associated with land life surveillance and the context generated by data are given to address these issues. The Wireless Sensors Network (WSN) and Artificial Intelligence (AI) give the option of monitoring fast landslides in real-time conditions. A proposed system in this paper shows real-time monitoring of landslides to preternaturally inform people through an alerting system to risky situations.

## 1. Introduction

Every year in nearly every region, hundreds of landslides erupt. Landslides occur increasingly often because of numerous factors, such as climate change, human activity, and topographic features [1]. The events normally arise during a big rain when the groundwater is transformed as a historical state by several factors. In rare situations, landslides suddenly occur without notice and are impossible to foresee and anticipate. To follow variations of insignificant elements for the aim of the prediction and to promptly identify the landslides, continual monitoring is essential. Hill pathways may harm structures nearby [2]. Landslide monitoring is primarily intended to safeguard individuals and these structures. A model can cover a huge region where landslide is possible with existing technologies. A system cannot be deployed in all risky places, so that inhabitants and traffic zones are protected [3]. Roads and buildings are becoming key items in highland and hill locations. In addition to ideas for improving the subsurface characteristics of the slope, it is another goal of the monitoring activity to find slides promptly and correctly.

The use of WSN has significant critical medical capabilities, while facing catastrophes like landslides and artificial intelligence is among the most powerful social deployments in alerts about environmental or man-made tragedies. WSN can operate large-scale, with low maintenance, scalability, flexibility, etc. [2, 3]. While WSN has its constraints, such as low memory, power, and bandwidth, its ability to be operated in hazardous conditions and low maintenance requirements makes WSN one of the finest real-time monitoring systems. Many artificial intelligence systems in the seismic analysis have been widely used during the past two decades. The major benefits of artificial intelligence approaches are their accurate quantitative base, their repetitiveness, their capacity to assess the impact of elements, and their capability for ongoing upgrading in a quantifiable manner [4]. Wireless sensor networks are the Earth's predictive system.  Figure 1 is the integration of a variety of sensors, wireless nodes, servers and gateways, and AI prognosis [5]. It is integrated into the design of the landslide-prone hill slope for constant monitoring of landslide with parameters that affect landslide factors, tiltmeter, dielectric moisture sensors, geophones, tension gauges, and piezometers sensors [6]. The strategic location of wireless nodes is to create a unified wireless mesh network to send sensor information to the computer through wireless intermediate nodes. The proposed model of landslides using AI is represented in Figure 1.

## 2. WSN System

The AI landslide prediction algorithms are used to monitor, test, store, and display data from these wireless nodes linked with multiple sensors and to provide the locally elected agencies and local people with audio-visual, Short-Mail (SMS), and e-mail alerts through the prediction of the incipient landslides. The power source of wireless nodes is replenished using the Solar Panel in the system design [7, 8].

### 2.1. Literature Survey

In Giorgetti, A [1], in this approach, geological sensors and camera sensor networks are used. Whenever the node value passes a given threshold, the camera sensor and the pictures are moved to the remote center. The sensor is activated. However, in our instance, the sensors are used using the boring hole technique and embedded under the ground by a range of sensor columns with a 30 m deep depth. The exactness of measurements for pore pressure and subterranean motion is enhanced without camera utilization due to a large number of intelligent devices. Kanungo et al. [2] discussed a setup of landslides telescope in Pakhi Landslide in Garhwal Himalayas, India, for the monitoring of land deformation and hydrological factors in real-time. The goal was to identify the mechanics of the motion of the tribulation. Such a method is expensive and unreasonable. However, a precipitation-based alerting threshold may be set, and a warning system can be sent depending on this amount of Automated Weather Station units (AWS). Suryawanshi and Deshpande [3] implemented different sensor kinds, including talks on different wireless sensor networking approaches for continuous landslide-risk monitoring of hazardous locations. The study includes many networking interfaces to communicate with ZigBee, WI-FI, and other distant analytics centers. GSM module is also incorporated in certain systems to transmit a high alert message to residents in the vicinity.

Wei Chen [5] discussed the latest generations, with the consequences of landslide risks increasingly serious, landslide prevention, and mitigation research receiving wide-ranging attention in important fields. The capacity to anticipate groundwater vulnerability, which may be utilized for designing land and urban planning in hilly locations, has been a major study issue. Xudong Hu [7] examined the possible use of landslide evaluation stacking ensemble learning techniques. SVM, ANN, LR, and NB, in addition, were chosen as basic students for the ensemble stacking technique. To assess the relevance levels of these basic students, the resampling technique and Pearson's analysis were employed simultaneously. Vu Van Khoa [8] described a wireless network sensor system (WSN) to detect catastrophes in remote locations. The design comprises three components, the Local Node System (LSNNS), the Cloud System (CS), and the Host System (HS). We have built up a suitable management program in which the HS gathers several data kinds in groups to monitor the field status and condition of nodes' remote location: node, node, LSNNS, and LSNNS data. HS and CS may be handled using analogous lists. The following were among the most prevalent types of landslides that arise [9] rotational landslides, are a concave upward curve (spoon shape), and are present on the surface of rupture, and the sliding motion is more or less rotating, and translational landslides are the bulk of soil and rock travels outward or down and outward, with minimal rotary motion or backward inclination; at this location, topple is a piece of rock that tilts or rotates forward and falls, bounces, or rolls down the hill. The Wireless Sensor Node translates the analog data from the sensor into quantitative information needed to make it legible by the machine. Moreover, this data is conveyed to the gateway. The microprocessor for an IEEE 802.15.4*e*-based wireless sensor network consists of the Wireless Transceiver, power supply, unit for power saving, and a Microcontroller collecting analog signals from sensors [10]. The software in the microchip enables the sensor nodes to connect for any node placed near the inside of the monitored region with self-organizing features. The connected device analyzes the information taken and transfers them using the hopping technique to another sensor node [11]. The surveillance data is handled by multiple networks during the transfer process to reach the gateway station after multi-hopping.

Landslide is a highly complex impacted by several causal elements comprising rainfall, seismic activity, weathering, humidity dynamic, PWP, water drainage and slope motions, etc. Landslide is a complicated occurrence. Many remote sensing technologies for landslide monitoring are now in place using satellite surveillance [12]. The major benefit of such approaches is that huge regions with high spatial resolution and 3D capabilities may be surveyed. Methods for remote sensing are good for mapping vulnerabilities, mapping risks, and postcatastrophe mapping, but they are restricted to real-time monitoring, which involves long-term revisits by the satellites [1, 13]. Seismic, Electromagnetic, Land Penetration Radar, and Electric Resistivity Tomography are a few of the noninvasive geophysical technologies used to track huge volumes of subsurface areas. However, these techniques are circuitous and lead to several nonsingle responses that restrict their use in trustworthy alerts [14]. Landslide surveillance procedures focused on geotechnical equipment such as extensometers, slope, and piezometers that permit precise measures, but these measurements are confined to the tiny regions on which the device is mounted. Systems focus on instruments that can still be utilized for major arteries and have a regional monitoring restriction. These are extremely difficult and expensive approaches; they involve heavy-duty, unmanageable technology, and efficiency at maximum, and therefore, they can truly be utilized in advanced detection [15].

#### 2.1.1. Recent Literature

In a recent article [16], the authors have elaborated a survey model by searching all possible ways of landslide detection using different approaches such as images and susceptible assessments where most of the potential landslides are predicted within remote location. But extraction of images is a difficult task, and it cannot be solved using assessment procedures. Therefore, after longsighted survey model, the authors [17] have integrated a software for searching and finding all hidden sights with low probability of failure. However, more errors are acquired in this type of landslide detection and natural language programs are combined with prior knowledge on system identification. By expanding the software model, a python program has been simulated [18] to analyze all shallow landslides in a particular area, where, in case of heavy rainfall, a control mechanism can be induced. As a new technology, a mapping technology, which is susceptible to distinct environmental aspects, has been reported [19], which is quite conceding model with high parametric evaluations.

### 2.2. Research Gap and Motivation

On the other hand, Early Warning System (EWS) is a cost-effective and extensively used early warning system model based on rainfall thresholds. Nevertheless, these cautions are sensitive to a wide range of false positives and do not offer any good solution either because there is not enough relevant information or owing to the lack of thin grain precipitation data in spaces and times. Area alerts are very general and may be adjusted to make them useful for a particular location and need a large number of years of precipitation measures to match the landslide incidents [16–21]. Rainfall thresholds are highly broad. In addition, monitoring one important landslide parameter is not adequate to resolve with confidence the requirement for early warning of landslides.

### 2.3. Objectives

The major aim is to build very precise sensor measurement techniques and a WSN multisensor system for collecting different parameters, including PWP, soil humidity, ground-based vibrations, and rainfall for precise, site-specific early warnings. A method based on data was used to ensure that early warnings are sufficiently trustworthy, reliable, and appropriately advanced. On multiparameter data, AI algorithms are incorporated with following constraints,

- Based on rainfall and PWP sensor data, you will arrive with a 24-hour prediction of slope stability circumstances.
- Learn from the past and make predictions about the current circumstances on the slope using statistical data.

The AI algorithms have made it possible to anticipate the path's real-time terms, so that robust systems may be designed during disasters when accurate data are not available. Another benefit of AI being integrated into multisensor data is that information may be utilized as a virtual sensor after understanding the path circumstances for a few years, whereas the actual sensors are reusable at other sites for renewal. In comparison with genuine WSN system data, all early cautions 24 hours before inclination stability and real-time sensor forecasts are all validated.

## 3. Data Management Center: A System Model

The method used ensures continuous sensor data transfers throughout the sensor nodes to the data management center (DMC). The DMC includes a database server and a scanning unit that analyzes, models, and simulates data on the ground to assess the possibility of a landslide. The information on the network is transmitted in real-time and the data analysis findings. Notifying services such as email, SMS, and MMS will be added to alert experts to the risk of landslides, network status, and system component monitoring [12]. The broadband or GPRS connection on the DMC provides the capability for the upload of real-time information straight onto a web page. The whole system is designed to monitor the residual recharging capacity and solar charge rate constantly. The technology also analyzes all wireless and geological sensors to detect defective nodes and sensor systems [13]. A feedback mechanism alters the sample rate of geophysical sensors continuously, compared to the climate differences in real-time.

WSN data is processed in real-time by the Data Management Center, which is located on the WSN field.

- Rainfall Intensity and Duration Limits.
- The slope's factor of safety (FoS) is an important consideration.
- Tilt and vibrations caused by movement sensors are recorded.

When the slope angle, soil properties, and PWP values at a given location in the sloppy region are combined, this function indicates the stability conditions of the slope and may be calculated. This statistic is represented as a nondimensional grid [12, 13]. The FoS of the Iverson model is defined in (1).

(1) $$\begin{array}{c} Fos=F_{g}+F_{j}+F_{d}=1. \end{array}$$

Here, *F*_*g*_ is a factor in a slope, *F*_*j*_ is a hydrogeologic factor, and *F*_*d*_ is a factor in soil cohesiveness and is shown in equations (2)–(4):

(2) $$\begin{array}{c} F_{g}=\frac{\tan\;\theta }{\tan\;\beta }, \end{array}$$

(3) $$\begin{array}{c} F_{j}=\frac{-PWP\;\left(S,t\right)\rho_{j}\tan\;\theta }{\rho_{r}S\;\sin\;\beta \;\cos\;\beta }, \end{array}$$

(4) $$\begin{array}{c} F_{d}=\frac{d}{\rho_{r}S\;\sin\;\beta \;\cos\;\beta }, \end{array}$$

where *θ* is an angle of soil friction, *β* is an angle of the slope, *d* is soil cohesiveness, *ρ*_*r*_ is the weight unit weight averaged in the depth of the soil, and *ρ*_*j*_ is the unit weight of groundwater. The rapidly adjusting factor in this equation is the PWP(S,t) variation of the pressures head, terms like as *d*, *ρ*_*r*_, *θ* are determined by soil test in the field, and the terms *β*, *ρ*_*j*_ are constants. When PWP grows in the soil, the efficient stress decreases, and strength in the soil is reduced [1]. FoS defines the slope failure, which is distinguished by the ratio of gravitational pull from the downhill to PWP's resistant stress. Ideally, if the ratio is 1, the two forces are balanced.

### 3.1. Constraints

If the level of FOS exceeds 1, that is, FoS >1, thus, the stress state in the soil exceeds that of the gravity; therefore, the slopes are stable at this depth. The stress-strain reduces when PWP is larger. If the FoS level is less than one, that is, if the FoS level is less than one, the slope is more likely to collapse at the depth. When calculating the depth of each susceptible site in our landslide early warning system, we use the real-time door pressures of the piezometers put in this specific spot to calculate the FoS at each vulnerable point at different depths. The real-time system can continue to collect such information and analyze the FoS variance of adaptively different pores in real-time [14]. The FoS is the indicator of the upcoming landslides. The cumulative FoS values from several slope locations are often used to assess the entire slope's sturdiness.

### 3.2. Sensors for Landslide Detection: Parametric Model

This paper was essentially intended to determine the sensors necessary to monitor and detect landslides. The selection of the right geotechnical sensors needs a deep understanding of the landslide phenomena, landslide characteristics, and distribution hydrological. The selection of the right geotechnical sensors needs a deep understanding of the landslide phenomena, landslide characteristics, and distribution hydrological. Forced landslides often occur following heavy, high-intensity, or lengthy medium-intensity rains in landslide-declined regions. Under heavy precipitation, rain penetration on the slope creates unstable decrease in the safety margin; transitory pores, a change in water table height, decrease in soils or climb force, rise in soil weight, and decrease in the angle of the rest [10–12]. These are resources to produce when the rainfall intensity exceeds the sloping hydraulic saturation conductance. The changes that occur in humidity, pores, rainfall, motion, and tremors inside the ground are the most important physical phenomena to be observed to prevent early warning of landslides. Following lengthy analysis, the geophysical sensors were chosen and utilized to analyze these phenomena [1].

(i) Dielectric moisture sensors: soil moisture sensors of the capacity type that detect the dielectric properties or permeability of the ground in which it is embedded were chosen.
(ii) Pore pressure piezometers: with increasing rainfall, rainwater collects in the holes of the soil and exerts an adverse strain that loosens the strength of the soil [2, 3]. So, it must be measured using the swinging wire piezometers or the strain gauge type piezometers, to detect groundwater hole stress.
(iii) Strain gauges: a pressure gauge is being used to monitor the motion of the soil layers by attachment to a DEP. Defaults of 0.5 mm per meter must be identified in the Deep Earth probe (DEP) [5]. For installation, strain measurements were utilized with varied strengths, such 100 X, 350 X, and 1000 X.
(iv) Tiltmeters: tiltmeters are used to measure motions of the soil layer like an extremely gradual creep or abrupt moves. For this situation, high-precision tiltmeters are necessary.
(v) Geophones: the geophone is used to analyze the landslide tremor. Landslide features need frequency assessment up to 250 Hz. The precision should not exceed 0.1 Hz, and these observations must be taken in real-time [8].
(vi) Rain gauges: the influence of precipitation on the slope, as well as the depths of the main groundwater or the increase of mass in the soil layer and the reduction in the stability of soil and rock, which may cause a landslide, is likely to change soil suction and positively pressure gradients [4, 5]. Using a tipping bucket, the rainfall intensity is 5,000 mm per year. A tipping bucket-type cordless rain gauge was utilized for placement where the tipping occurrence is recorded as 0,001.
(vii) Temperature sensors: as for the temperature, the physical features of soil and groundwater change. The 1/10th degree precision Celsius recorded is adequate for each 15 min.
  (5) $$\begin{array}{c} \text{MSE}=\frac{1}{G}\overset{G}{\underset{j=1}{\sum }}{\left(x_{i}-\hat{x_{i}}\right)}^{2},\\ \text{RMSE}=\sqrt{\frac{I}{k}\overset{k}{\underset{i=1}{\sum }}{\left[\left[h\left(b_{i}\right)-y_{i}\right]\right]}^{2}}, \end{array}$$

where *x*_*i*_ is predicted responses, $\hat{x_{i}}$ is observed responses, respectively, and *G* is the total number of variables.

(6) $$\begin{array}{c} \text{ACC}=\frac{\text{TP}+\text{TN}}{\text{TP}+\text{TN}+\text{FP}+\text{FN}}\;\times \;100\%,\\ \text{Sensitivity}=\frac{\text{TP}}{\text{TP}+\text{TN}}\;\times \;100\%,\\ \text{Specificity}=\frac{\text{TN}}{\text{TN}+\text{FP}}\times \;100\%. \end{array}$$

All geophysical sensors listed above are fitted to wireless sensors that can detect with little operation in real-time where the necessary values can be detected using the abovementioned corresponding values.

### 3.3. Data Acquisition Modules

This section is required to gather data from geophysical sensors, both analog and digital. The DEP data gathering model is integrated (Deep Earth probes). This layer receives the digital information from the numerous sensors utilizing the digital drivers [13]. For data processing from the sensor circuits and stimulation circuits, analog drivers are used. Different data sources have been compiled to identify ancient occurrences in the area, historical data obtained by the Civil Defense Authority, national reports, and surveys with residents [22]. Large and complex surveillance applications require upcoming events and the management of the caches of every node to prevent loss of occurrences and data. The data analysis unit is the fundamental aspect in which all input and output signals in the wireless sensor nodes may be processed [15]. The primary features of these modules are to plan the occurrences and manage caches in a distributed system. Four essential features have been added to the routing:

- Sensor sampling: this unit is required to assist clear communication through specialized coupling circuits between geophysical sensors and the connected wireless sensor node. It can source and gather data from geophysical sensors at the intersample rate set by the user. This is subsequently forwarded to the module for buffer management [19].
- Health monitoring: this unit monitors the condition of the remote system and nodes. The node health feature gives the power status in the node, the battery life, and other things needed. The health network feature is employed by regular upgrading of the neighborhood addressing to detect nodes dead in the network. These neighborhood addresses are utilized to route data to the gateway of the probe efficiently [10, 11].
- Power saving: this component gives the wireless sensor nodes with power conservation techniques. The changes to a remote system node-like ‘sleep,' ‘monitor,' ‘active,' and ‘off' are integrated. The integration of geophysical sensor state transitions could further increase power efficiency [20]. Thus, the precision values can be calculated using the following equations:

(7) $$\begin{array}{c} \text{Precision}=\frac{\text{TP}}{\text{TP}+\text{FP}}\;\times 100\%\;,\\ F=\frac{2*\text{Precision}*\text{Sensitivity}}{\text{Precision}+\text{Sensitivity}}\times 100\%. \end{array}$$

## 4. Optimization Using AI

Three different types of artificial intelligence algorithms have been selected to assess the viability of using artificial intelligence in landslide analysis and tracking [15]. The use of artificial intelligence techniques has several benefits as they can adapt their inner structure to current landslide information. In addition, the AI is having the ability to automatically extract information from big datasets. In an attempt to include a precise landslide method, the frameworks are cost-efficient and quicker than traditional models and can be lengthened to broad area analyzes. They are capable of supervised learning (projections of continuing factors). Their frameworks are more cost-effective than standard models [16]. In this paper, the landslide monitoring was carried out using three advanced AI approaches, which differ in complexity. To assess their effectiveness, SGDA, LR, and SVM are included, and they are discussed below.

### 4.1. Stochastic Gradient Descent Algorithm

The technique of stochastic gradient descent (SGDA) is a dramatic reduction approach, which uses a tiny randomly chosen subset to calculate the optimization problem gradient. The batch size is referred to in one cycle as the quantity of the classifier [17]. Through the short batch size of the variables, the convergence may be changed more often than the gradient descent. The highest update frequency and the simpler perception-like method are available with batch size 1, in extreme situations. The weights of the functionality are changed in the SGDA with the given (8) for the classifier:

(8) $$\begin{array}{c} R^{y+1}=R^{y}+\beta_{y}\frac{\delta }{\delta R}\left(K\left(i,R\right)\right)-\frac{P}{Q}\sum_{g}\left|R_{g}\right|, \end{array}$$

where *Q* is the batch size, *P* denotes the meta-parameter that regulates the degree of regularization, *R* denotes the iteration counter, *β*_*y*_ denotes the learning rate, *R*_*g*_ denotes the weight of the feature, and *L*(*i*, *R*) denotes the conditional log-likelihood of the ith training sample.

### 4.2. Logistic Regression

A prominent numerical method utilized for measuring the vulnerability of landslides is logistic regression LR. It provides a multidimensional connection between independent and dependent variable regression. Circular, periodic, or both variables might be used [15, 16].

By taking the highest chance value, the LR algorithm calculates the probability of a given landslide occurrence. The dependent variable is a data point in the case of landslide prediction (landslide and non-landslide). The LR algorithm may be stated as follows:

(9) $$\begin{array}{c} A=\frac{1}{1+e^{-h}}, \end{array}$$

where *A* is deﬁned as the probability of a past landslide event, and *f* is determined by

(10) $$\begin{array}{c} h=b_{0}+b_{1}z_{1}+b_{2}z_{2}+\cdots +b_{n}z_{n}, \end{array}$$

where *n* is the total number of factors, b0 is the application's intercept, bi, *i* = 1,2,…, *n* is the application's slope coefficient, and *z* = *z*_*i*_, *i* = 1,2,…, *n* is the characteristics of the factors.

### 4.3. Support Vector Machine

A prominent categorization method presented in the 1990s also includes a support vector machine. It is regarded as one of the more flexible techniques in many contexts for its great result [18]. A vector supporting machine utilizes cores to extend the function space and to measure the similarity between two observations to reflect the nonlinear supervised classification limit. (11) defines, for instance, a popular core called the radial kernel.

(11) $$\begin{array}{c} U\left(d_{j,}d_{\dot{\dot{j}}}\right)=\exp\left(-\theta \sum_{i=1}^{p}{\left(d_{ji}-d_{\dot{j}i}\right)}^{2}\right), \end{array}$$

where *d*_*ji*_ and *d*_*j'i*_ are the jth pair of observations of the ith predictor, *p* is the number of predictors, *θ* is a tuning parameter that accounts for the smoothness of the decision boundary, and *U* stands for the kernel function. The flow chart of SVM for landslide detection is deliberated in Figure 2.

## 5. Outcomes

Validation is essential in the course of landslide monitoring. Various statistical techniques have been taken to evaluate them, but the conventional verification standards are still under dispute [19]. The sensitivity, specificity, ACC, the F, the MAE, and RMSE were used for prediction evaluations.  Table 1 presents the tolerances and VIFs for the 5 landslide conditioning factors in this paper. The analysis shows that the VIF value maximum is 2.768, and the tolerance maximum is 0.456. It meets crucial values (tolerance >0.1 or VIF <10) and shows that no multicollinearity is present with five landslide conditioning parameters as shown in Figure 3.

This analysis revealed that landslide monitoring is possible with artificial intelligence (LR, SVM, and SGDA).  Figure 4 reveals that the highest proportion in the region is LR (58.90%), trailed by the highest grade (29.90%), high (5.89%), low (4.78%), and moderate (3.45%). As far as SVM is concerned, Figure 3 indicates that the highest area rating is extremely low (54.78%), trailed by a very large area (29.78%), high area (6.90%), low area (4.89%), and moderate area (4.78%).

As for SGDA, it appears in Figure 4 that the greatest range of the very low class (51.34%) is followed by the high (26.01%), high (9.43%), low (6.45%), and moderate (6.23%) classification as shown in Table 2.

Table 3 provides three techniques' system performance. The results show that, in the case of the landslide function approximation (Sensitivity = 92.76%), the LR method shows the highest performing effect, trailed by SVM (Sensitivity = 77.67%) and SGDA (Sensitivity = 84.78%). In contrast, the results showed that the LR method had the highest accuracy values (93.78%). The highest F measurement was 0.95, the lowest MSE was 0.045, and the lower MSE was 0.126 as shown in Figure 5.

## 6. Conclusions

This disaster is one of the biggest and most dangerous in the Earth. Using wireless sensor data, we have built artificial intelligence systems that can accurately predict sliding movements. It is possible to provide real-time and continuous monitoring of different prominent landslide factors, such as precipitation, vertical and horizontal mass inclination of rock, and displacement of rock and soil water in structures, utilizing the wireless sensor network for landslide prediction. The main goal of this paper is to analyze and evaluate three advanced artificial intelligence landslide surveillance technologies, that is, LR, SVM, and SGDA. These methods were evaluated in terms of their success. The accuracy of 93.78 percent shows that LR models are very competitive. In the future, we planned to use deep learning techniques.

## Figures and Tables

**Figure 1:** Landslide monitoring using wireless sensors and artificial intelligence.

**Figure 2:** SVM for landslide detection using kernel functions: the proposed flow.

**Figure 3:** Conditioning factors. (a) Slope angle. (b) Slope aspect. (c) Altitude. (d) Curvature. (e) Rainfall.

**Figure 4:** Percentage of susceptibility classes. (a) LR. (b) SVM. (c) SGDA.

**Figure 5:** Performance metrics.

**Table 1:** Multicollinearity diagnosis of landslide conditioning factors.

Factors	Collinearity statistics	
	Tolerance	VIF
Slope angle	0.799	1.176
Slope aspect	0.689	1.780
Altitude	0.456	2.768
Plan curvature	0.675	1.499
Rainfall	0.411	2.458

**Table 2:** Percentage of different landslide monitoring classes.

AI model	Very low	Low	Moderate	High	Very high
LR	58.90	4.78	3.45	5.89	29.90
SVM	54.78	4.89	4.78	6.90	29.78
SGDA	51.34	6.45	6.23	9.43	26.01

**Table 3:** Model performance.

AI model	MSE	RMSE	Accuracy	Sensitivity	Specificity	*F*-measure
LR	0.045	0.126	93.78	92.76	99.78	0.95
SVM	0.167	0.345	84.89	77.67	96.87	0.84
SGDA	0.234	0.378	86.78	84.78	93.12	0.83

## Data Availability

The datasets used and/or analyzed during the current study are available from the corresponding author upon reasonable request.
